The article "Sports Video Athlete Detection Based on Associative Memory Neural Network" was retracted in 2023. Reasons: signs of a paper mill; suspected computer-generated content; unreliable results or conclusions; concerns about the data.

# Sports Video Athlete Detection Based on Associative Memory Neural Network

**DOI:** 10.1155/2022/6986831

**Published:** 2022-02-15

**Authors:** Jingwei Yang

**Affiliations:** ^1^School of Physical Education, Xinyang Normal University, Xinyang 464000, China; ^2^School of Physical Education, Central China Normal University, Wuhan 430079, China

## Abstract

Aiming at the detection of athletes in sports videos, an automatic detection method based on AMNN is proposed. The background image from the image sequence is obtained, the moving area is extracted, and the color information of pixels to extract the green stadium from the background image is used. In order to improve the accuracy of athletes' detection, the texture similarity measurement method is used to eliminate the shadow in the movement area, the morphological method is used to eliminate the cracks in the area, and the noise outside the stadium is removed according to the stadium information. Combined with the images of nonathletes, a training set is constructed to train the NN classifier. For the input image frames, image pyramids of different scales are constructed by subsampling and the positions of several candidate athletes are detected by NN. The center of gravity of candidate athletes is calculated, a representative candidate athlete is obtained, and then, the final athlete position through a local search process is determined. Experiments show that the system can accurately detect the motion shape of moving targets, can process images in real time, and has good real-time performance.

## 1. Introduction

Detecting and tracking athletes in sports videos can provide important information for high-level sports video processing, such as motion analysis, event detection, and 3D reconstruction [1, 2]. Attaching various sensors to athletes and then acquiring data through sensors are the traditional method of detecting and tracking athletes. These methods, on the other hand, place additional constraints on athletes and have a negative impact on their normal performance [3]. As a contactless method, the video-based athlete detection and tracking method developed in recent years have been widely studied and applied [4].

It is of great significance to detect and track athletes in sports videos, which is conducive to various higher-level processing of videos, such as adding automatic explanation function to videos, quick retrieval of important events in videos, and tactical analysis of videos [5, 6]. Moving target detection and tracking mainly involve the knowledge of image processing, pattern recognition, computer vision, artificial intelligence, and other disciplines, in many fields. For example, human-computer interaction, video surveillance, traffic management, and content-based video retrieval have wide application prospects and potential economic value [7]. Therefore, researchers have been inspired to do a lot of research on it, and many different methods have been put forward. Another important direction in sports video analysis is the detection of exciting events. Segmentation and tracking of sports videos can assist the detection of exciting events, as well as semantic and strategic analysis. We can judge the detection of some specific events through target detection and tracking analysis. In this paper, the neural network (NN) technology [8, 9] with associative memory (AM) function is studied. And, a sports video athlete detection model has been put forward based on associative memory neural network (AMNN).

Digital video technology has been developed and popularized in tandem with scientific and technological advancements. It is now possible to obtain various types of videos through various channels, thanks to increased network transmission bandwidth and lower costs of various hardware devices [10]. Computers can now execute various complex algorithms, thanks to increasing storage capacity and computing power [11]. These technological and equipment advancements lay the groundwork for future image processing and video analysis systems research and development. The focus of these people's attention to sports video also focuses on sports targets, balls, or players. Detecting athletes' areas in sports videos is the premise of tracking athletes [12]. The application based on AMNN can extract athletes' trajectory and other information from the game video, which can help coaches analyze players' behaviors and study opponents' strategies and weaknesses. Based on the analysis of the current main moving target detection and tracking algorithms, this paper focuses on the methods of detecting and tracking athletes in sports videos and improves the traditional moving target detection and tracking algorithms. Aiming at the characteristic that AMNN is easy to fall into local minimum, particle swarm optimization is introduced to optimize the network weights, and a network with high convergence performance is obtained. A prototype system is developed to verify the effectiveness of the algorithm.

## 2. Related Work

The athlete detection algorithm based on middle-level feature blocks and the athlete segmentation algorithm based on superpixel classification are realized in the literature [13, 14] based on a detailed analysis and summary of the characteristics of sports videos and related rules. The literature [15] proposed a method for detecting the stadium area by obtaining the stadium's adaptive color. A method to automatically extract the venue color in sports videos was proposed in the literature [16, 17]. It uses a Gaussian mixture model to calculate the parameters with an algorithm, which is different from previous studies, and the experiment is similar to the previous one. The Kalman filter models each pixel and tracks its change in the literature [18, 19]. This method can handle scene lighting changes, but it becomes invalid when new objects are added to the scene or the original objects are removed. For the detection of multiscale athletes in sports videos, literature [20] proposes an automatic detection method based on CNN. The literature [21] describes the function realization and concept of AM in detail, as well as the drawbacks of having to use a binary input signal in practice. By combining the advantages of strong nonlinear processing of BP networks with the advantages of fitting the network structure reasonably, the network structure can be widely used in practice. The dynamic method based on prediction is used to model the dynamic scene in literature [22, 23]. This method can deal better with light changes and subtle movements in the scene, such as water waves and branches swinging, but it requires a large number of images without moving objects to train the model. A key pose extraction system for weightlifting video was designed by literature [24]. A display module and a key frame extraction module are included in the system. The key frame extraction module includes feature extraction and key frame extraction of weightlifting video frames, while the display module includes video playback and key frame display. Literature [25] uses the Gaussian mixture model to model every pixel in the scene and updates the model in real time by the online approximation method, which can reliably deal with the situation of illumination change and disturbance of chaotic motion in the scene. At present, the commonly used tracking methods include model-based tracking, region-based tracking, and feature-based tracking. Literature [26] studied discrete Hopfield NN and discussed the structure and the theory of convergence stability in detail. The continuous adaptive mean shift algorithm proposed in literature [27] uses the color features of objects to track irregularly moving nonrigid objects in video frame sequence quickly and robustly. Literature [28] uses the combination of adaptive Gaussian mixture model and CamShift algorithm to detect and track players in badminton video. In this paper, a method of moving object detection in sports video based on the AMNN model is proposed. The experiment shows that the system can accurately detect the motion shape of moving targets, process images in real time, and has good real-time performance.

## 3. Methodology

### 3.1. AMNN

Artificial neural network (ANN) is an information processing system that simulates the structure and function of a simplified biological NN and abstractly utilizes some basic characteristic theories. This network receives external information through vision [29], smell, and taste, processes it in the brain, and then outputs signals through the executive organs, thereby forming a system with the characteristics of a closed-loop control system.

Humans can study ANN in the same way they can study the various functions of the human brain. Distributed storage and fault tolerance, large-scale parallel processing capabilities, self-learning, self-organization and adaptability, and the ability to handle complex systems are all features of ANN [30]. AM is a key component of NN theory, as well as a key function of NN in intelligent control, pattern recognition, and artificial intelligence. It primarily makes use of NN's high fault tolerance, which allows it to reconstruct incomplete, defaced, and distorted input samples into a complete prototype suitable for identification, classification, and other purposes.

The Hopfield network, also referred to as the AM network, is a type of computer network. Hopfield network is a typical single-layer feedback NN, with rich dynamic behavior, simple structure, and higher computing power when compared to other networks. A discrete-time system is a discrete Hopfield neural network (DHNN). A weighted undirected graph can be used to show it. Every node has a threshold, and each side of the graph has a weight. The graph's order corresponds to the network's order. As a standard network for classification tasks, NN will typically add a fully connected layer and a classifier to the final layer. During the training process, a dropout operation is added to the fully connected layer to prevent overfitting, and the output value of the node is randomly set to 0 to prevent overfitting. Although this slows down training, it effectively prevents overtraining. The basic structure of the Hopfield network is shown in Figure 1.

The network weakens the false state by adding an additional attractor to improve the fault tolerance of the network. Because one of the fundamental problems of Hopfield is that in addition to the existence of attractors with memory samples, there are also “redundant” stable states, that is, the existence of pseudo-states. The existence of pseudo-states affects Hopfield's fault tolerance. If the pseudo-states can be reduced or even eliminated, the attraction domain of the state can improve the fault tolerance of Hopfield and increase the memory capacity. Because the neurons in the Hopfield network are connected to each other, this fully interconnected way makes the output of each neuron in the network feedback to the input of other neurons at the same level, so the network has no other external input. Under these circumstances, it can also enter a stable state.

The learning process of DHNN, like that of other NNs, is the formation of a network connection weight matrix. Hopfield is a constantly changing system. Once the network's connection weight matrix is learned and formed, as long as a specific pattern sample is input, the network will continue to evolve until the system reaches the state space's steady state. This steady state is the network's output state, or the input vector's associative memory output. After the network has been trained, it can be run with an initial input *X* to determine the network's initial output state. This state is fed back to the input terminal and used as the input signal for the network processing stage's next iteration. Because the network takes a certain amount of time to transmit and process information, the two input signals may differ before and after the new input gives birth to the next output. The network's operation process, or the repeated feedback process, is an example of such a cycle. If the network is stable, the change in the output state of the network will decrease as the network runs with multiple feedbacks until it no longer changes and reaches a steady state.

### 3.2. Detection and Tracking of Moving Objects in Sports Videos

The so-called moving target tracking is to detect each independently moving target or region of interest to users in each frame of images and locate these targets or regions in subsequent frames. In practical application, tracking the moving target is very important. By tracking the moving target, we can get its motion parameters, such as position, velocity, and acceleration, which not only helps to calculate the motion trajectory of the moving target but also provides a reliable data source for the motion analysis and scene analysis of the target in the scene. Sports videos have different characteristics of different lens types, which can provide prior knowledge for video content analysis. The video is divided into shot sequences by shot boundary detection, and the types of shots are detected; that is, the shots are divided into short shots, medium shots, and long shots. This series of processing before athlete detection and segmentation is called video preprocessing. The athlete detection process is shown in Figure 2.

There are three commonly used algorithms in motion detection research: interframe difference, background subtraction, and optical flow. The difference between the current frame and the previous frame image is calculated using the interframe difference method, which is suitable for a dynamically changing environment. However, it only extracts the part of the logo that moves in relation to the background; it is not a fully moving object. The optical flow method is used to detect the application logo's changing optical flow characteristics over time. Its advantage is that it can detect moving objects independently without prior knowledge of the scene, and it can be used while the camera is moving. The disadvantage is that the calculation is time-consuming and difficult. Real-time detection is difficult to achieve without the necessary hardware support. Background subtraction is the most common technique for separating moving objects from a scene, particularly when the scene is relatively stable. The background subtraction method's main idea is to compare the current image to the background image by using a reference image that represents the background. If there are differences in pixel features, pixel area features, or other features in the same position, these are motion areas, which may correspond to actual moving targets.

Before detecting and identifying the image, it is necessary to preprocess the image, try to eliminate the noise, improve the image quality, protect the trade information, reduce the calculation amount of subsequent processing, and improve the accuracy of processing. There are strong rules in shooting and editing techniques in sports videos, and the characteristics of different shots and the differences between different shots are obvious. In the telephoto lens, the competition field occupies the largest proportion, and the athletes are also concentrated on the competition field, so the competition field area is detected first, and after the athletes are detected, more accurate athletes can be obtained by using the uniform color of the sports field and removing the color of the sports field. In the middle shot, the field color still occupies a certain proportion in the image, and if the telephoto scene has been processed, the stored ground color is used to remove the nonathlete area of the image of the middle shot that belongs to the competition field part.

In order to achieve an accurate positioning effect, a local search process is performed on the area around the center of each candidate athlete in the image scale space. In the image scale space, a small search space focused on the position of the candidate athlete is defined, which corresponds to a small pyramid focused on the center of the candidate athlete. The pyramid covers a scale from 0.8 to 1.5 times the size of the candidate athlete. For each scale, the candidate athlete is marked with a 16 × 16 pixel grid around the center of the candidate athlete. Mutual information can measure the similarity between two things. If two things are more similar, the mutual information between them will be smaller; otherwise, it will be larger. For shots, the frame images inside a shot are very similar, but the frame images between different shots are quite different. Therefore, mutual information is considered to measure the similarity between two frames.

### 3.3. Construction of the Detection Model Based on AMNN

The model-based tracking method models the shape characteristics of the target object and then tracks the model in the image sequence. The extraction of moving targets, that is, on the basis of existing images, extracts the required foreground targets through image segmentation.

Because an object is sometimes not a whole after image segmentation, it will be divided into several parts, or an object will be divided into several close independent areas. This paper makes a copy of the segmented image, expands it, and then assigns a number to it. If the areas after the expansion are connected to form a whole, they are identified as a whole, and the whole is marked as a region to be detected on the original image. The tracking accuracy of a model-based tracking method is dependent on the accuracy of the target object's geometric model. The main state transformations for a rigid moving target during movement are translation, rotation, and so on. When tracking a moving target, this method can produce better results.

Suppose a group composed of *M* particles flies at a certain speed in the n-dimensional search space, and the state attributes of particle *i* in the *t*-th iteration are set as follows:

Location:
  (1) $$\begin{array}{c} X_{i}^{t}=\left(x_{i1}^{t},x_{i2}^{t},\ldots ,x_{in}^{t}\right),\\ x_{in}^{t}\in \left[L_{n},U_{n}\right]. \end{array}$$
*L*_*n*_ and *U*_*n*_ are the lower limit and upper limit of the search space, respectively.
Speed:
  (2) $$\begin{array}{c} V_{i}^{t}=\left(v_{i1}^{t},v_{i2}^{t},\ldots ,v_{in}^{t}\right),\\ v_{in}^{t}\in \left[v_{\min,n},v_{\max,n}\right], \end{array}$$
where *v*_min,*n*_ and *v*_max,*n*_ are the minimum and maximum speeds, respectively.
Individual optimal position:
  (3) $$\begin{array}{c} P_{i}^{t}=\left(p_{i1}^{t},p_{i2}^{t},\ldots ,p_{in}^{t}\right). \end{array}$$
Global optimal position:
  (4) $$\begin{array}{c} P_{g}^{t}=\left(p_{g1}^{t},p_{g2}^{t},\ldots ,p_{gn}^{t}\right). \end{array}$$
Here, 1 ≤ *i* ≤ *M*. With the above definition, the iterative formula of the algorithm can be described as follows:
  (5) $$\begin{array}{c} v_{in}^{t+1}=wv_{in}^{t}+c_{1}r_{1}\left(p_{in}^{t}-x_{in}^{t}\right)+c_{2}r_{2}\left(p_{gn}^{t}-x_{in}^{t}\right),\\ x_{in}^{t+1}=x_{in}^{t}+v_{in}^{t+1}. \end{array}$$
Here, *r*_1_, *r*_2_ is a random number between (0, 1). *c*_1_, *c*_2_ is the acceleration factor. *w* is called the inertia weight, which determines how much the particle inherits to the current velocity. Appropriate value helps to balance search ability and development ability, and usually, a linear decrease method from 0.9 to 0.4 is used. The linear decreasing formula is
  (6) $$\begin{array}{c} w=w_{\text{start}}-\frac{w_{\text{start}}-w_{\text{end}}}{t_{\max}}\times t, \end{array}$$
where*t*_max_ is the maximum number of iterations; *t* is the current iteration number; *w*_start_ is the initial inertia weight; and *w*_end_ is the termination inertia weight.

Because the selection of threshold can't make all video frames have a better segmentation effect, when this paper intercepts the region of interest, more background information will be mistakenly regarded as foreground information. Mapping the detected pixel points of candidate athletes into the input image, the candidate athletes are grouped according to their distance in the image and scale space. Each group of candidate athletes is fused into a representative candidate athlete, whose center and size are the average of the center and size of each candidate athlete in this group. After the grouping algorithm is applied, a representative set of candidate athletes is obtained, which is used as the basis for accurately locating athletes and eliminating false positives in the next stage of the algorithm.

Occlusion between athletes and other objects is common in sports videos. In some videos, for example, athletes are blocked by the net, and there are various types of motion disturbances, as well as shadows. Because of the complexity of sports video, the detected motion foreground map frequently contains a lot of noise or has gaps in the motion area. To extract the athlete area more precisely in subsequent processing, the foreground image must be processed at the pixel level, removing noise, filling gaps, and eliminating shadows. Pixels are divided into boundary points and nonboundary points, with boundary points being classified as brighter or darker depending on the brightness of their surroundings. The gray level corresponding to the highest peak in the two histograms is used as the threshold, and the gray level corresponding to the highest peak in the two histograms is used as the histogram. This method is recursively applied to image system points whose gray levels are higher or lower than this threshold until a predetermined threshold number is obtained. In the iterative process, the centroid (*x*_*c*_, *y*_*c*_) of window *w* is as follows:

(7) $$\begin{array}{c} x_{c}=\frac{\sum_{x\in w}\sum_{y\in w}xP\left(x,y\right)}{\sum_{x\in w}\sum_{y\in w}P\left(x,y\right)},\\ y_{c}=\frac{\sum_{x\in w}\sum_{y\in w}yP\left(x,y\right)}{\sum_{x\in w}\sum_{y\in w}P\left(x,y\right)}. \end{array}$$

Resize the window to

(8) $$\begin{array}{c} s=2\times \sqrt{\frac{\sum_{x\in w}\sum_{y\in w}P\left(x,y\right)}{256}}. \end{array}$$

If only a fixed global threshold is used to segment the entire image when there are some situations in the image, such as shadows, uneven illumination, different contrasts in different places, sudden noise, and changes in background gray level, the segmentation effect will be affected because the situations in different parts of the image cannot be taken into account. To segment each part of the image separately, one option is to use a set of thresholds related to pixel positions. Athlete detection results based on middle-level feature blocks can provide polygonal areas of athletes in addition to rectangular box representation. To obtain more accurate segmentation results, the relationship between polygon domain representation and athlete contour is combined, using superpixels as the basic unit, marking the classification of superpixels according to the overlapping ratio of superpixels and polygon regions, and using the marking information and rectangular frames as interactive information.

## 4. Results Analysis and Discussion

In sports videos, athletes' movements are irregular, and their postures will change in various ways. The colors of athletes and scenes may be similar, and there is often mutual occlusion between athletes. In this paper, the obtained video is converted into a frame-by-frame video stream image as the system input. The system detects the input image, and if it is the first frame image, the image as the background is preprocessed and initialized the background model. Then, it is judged whether the input image is the second frame image, and if it is the second frame image, the image is preprocessed. The experimental results are shown in Figure 3.

Expansion is the process of merging the reasonable area in contact with the edge of an object into the object and expanding the boundary outward. If the number of expansions is too small, the lines forming the capture area are too thin to cover all possible ranges of soldiers, resulting in missing capture. If the expansion times are too large and the lines forming the capture area are too thick, the range of the capture area will be too large, which will increase the number of pixels searching for nonzero gray values and slow down the running speed of the algorithm. In further experiments, the detection speed of moving targets by different methods is compared, and the results shown in Figure 4 are obtained.

Noise and light sources often affect the sample points around the players, reducing their reliability. The farther away from the center of the athlete's area, the lower the pixel's reliability, and the greater the chance that the pixel is covered by other objects or belongs to the background. As a result, when calculating the histogram of the athlete area, it is reasonable to give different weights to pixels at different positions in the athlete area. The greater the weight corresponding to the pixel, the closer it is to the region's center, and vice versa. When the same video sequence is fast-forwarded at 4x speed under different quantization parameters, Figure 5 compares the number of transmission bits required by this method and the traditional method.

Even in the case of occlusion, the head of the human body still has obvious characteristics, so it is possible to divide multiple human bodies that are stuck or occluded into a single human body according to the characteristics of the head of the human body.  Figure 6 is a comparison result of moving object segmentation results by different threshold processing methods.

There is a lot of foreground noise in the picture, which will have a great influence on the detection results. Because the moving target is blocky and has a moving rule, the foreground noise appears sporadically, and the position is random. In the following moving target tracking algorithm, the foreground noise can be removed according to these features to get the accurate moving target.

We can compare the textures of the corresponding areas in the foreground area and the background image and judge whether the foreground area is a shadow or a real moving target according to the similarity of the textures. The verification of the detection range is extracted from the position coordinates of the correct moving target in the detection result, as shown in Figure 7.

It can be seen that this method is superior to the other two methods in detecting athletes in sports video. The other two methods and this method are also used to detect athletes. The comparison results of interference handling capabilities of these three methods are shown in Figure 8.

As can be seen from the data in Figure 8, this method has the best interference handling ability. This method provides a better tracking effect while also achieving the desired result. To fully realize the detection of moving targets, a frame of the system's input image will first undergo image scale transformation, filtering, and denoising through image preprocessing and then undergo the steps of image binarization, morphological processing, target edge detection, and so on. Finally, the blocks in the tracking area are merged based on adjacency and similarity, and a unified gray value is assigned, revealing the moving target's detected shape. Experiments show that the system can detect the motion shape of moving targets with high accuracy, process images in real time, and perform well in real time.

## 5. Conclusions

Motion detection and tracking are difficult fields of study. In this field, researchers have done a lot of work and have made some breakthroughs in theory and application. The key step in analyzing and processing sports videos is detecting and tracking athletes. This paper focuses on the methods of detecting and tracking athletes in sports videos, based on an analysis of the current commonly used methods of detecting and tracking moving targets. This paper proposes an AMNN-based method for moving object detection in sports video that takes full advantage of various technologies and processing means and outperforms previous inspection models. To address the issue of the model's learning rate being too slow in the early stages, the model's updating method has been improved, and the learning rate has been accelerated. The detection method used in this paper is more capable of dealing with slow changes in illumination in a dynamic background. Furthermore, different lens types in sports videos have distinct characteristics, and athletes who use the same lens type compete under the same set of rules. This paper summarizes these traits and rules and employs a middle-level feature block classifier to distinguish between different lens types and train different athletes to detect athletes in the video. Simulation experiments back up the method presented in this paper. The results show that the method presented in this paper has a wide detection range and strong interference processing ability. This scheme has a high rate of detection.

## Figures and Tables

**Figure 1:** Basic structure of the Hopfield network.

**Figure 2:** Athlete detection process.

**Figure 3:** Comparison of detection accuracy of three methods.

**Figure 4:** Comparison of detection speed of three methods.

**Figure 5:** Comparison of the number of bits to be transmitted in double-speed fast forward.

**Figure 6:** Comparison of segmentation results of moving objects by different threshold processing methods.

**Figure 7:** Verification results of the detection range of several methods.

**Figure 8:** Interference handling ability verification result.

## Data Availability

The data used to support the findings of this study are included within the article.
